# Selective enhancement of hypoxic cell killing by tempol-regulated suicide gene expression

**DOI:** 10.3892/or.2015.4020

**Published:** 2015-05-29

**Authors:** GO KAGIYA, RYOHEI OGAWA, RAJANI CHOUDHURI, JOHN A COOK, MASANORI HATASHITA, YOSHIKAZU TANAKA, KANA KODA, KEI YAMASHITA, MAKOTO KUBO, FUMITAKA KAWAKAMI, JAMES B MITCHELL

**Affiliations:** 1 School of Allied Health Sciences, Kitasato University, Minami-ku, Sagamihara, Kanagawa 228-8555, Japan; 2 Department of Radiological Sciences, Graduate School of Medicine and Pharmaceutical Sciences, University of Toyama, Toyama 930-0194, Japan; 3 Radiation Biology Branch, National Cancer Institute, National Institutes of Health, Bethesda, MD 20892, USA; 4 Biology Group, The Wakasa Wan Energy Research Center, Tsuruga, Fukui 914-0192, Japan; 5 Radiation Oncology, The Cancer Institute Hospital, Japanese Foundation for Cancer Research, Koto-ward, Tokyo 135-8550, Japan; 6 Graduate School of Medical and Pharmaceutical Sciences, Chiba University, Inage-ku, Chiba 236-8555, Japan

**Keywords:** tempol, hypoxia, HIF-1α, hypoxic cell killing, suicide gene, gene therapy

## Abstract

The presence of hypoxic regions within solid tumors is caused by an imbalance between cell proliferation and angiogenesis. Such regions may facilitate the onset of recurrence after radiation therapy and chemotherapy, as hypoxic cells show resistance to these treatments. We found that tempol, a nitroxide, strongly induces the accumulation of hypoxia-inducible factor (HIF)-1α, particularly under conditions of hypoxia. We, therefore, evaluated whether tempol enhances the gene expression via HIF-1α, potentially leading to various applications for cancer gene therapy targeting hypoxic cells. Consequently, following treatment with tempol under hypoxia, the luciferase (Luc) activity in the cells transfected with the plasmid containing the *luc* gene with the oxygen-dependent degradation domain and a promoter composed of hypoxia-responsive elements increased up to approximately 10-fold compared to that observed in cells treated identically with the exception of tempol. The plasmid constructed by replacing the *luc* gene with the *fcy::fur* fusion gene as a suicide gene, strongly induced the accumulation of the Fcy::Fur fusion protein, only when incubated in the presence of the hypoxic mimic CoCl_2_ and tempol. The transfected cells were successfully killed with the addition of 5-fluorocytosine to the cell culture according to the *fcy::fur* fusion gene expression. As similar but lesser enhancement of the Luc activity was also observed in solid tumor tissues in nude mice, this strategy may be applied for hypoxic cancer eradication.

## Introduction

Solid tumors are highly heterogeneous in terms of oxygenation and contain hypoxic cell regions as a result of an imbalance between cell proliferation and angiogenesis. As the primary cellular and systemic response to hypoxic stress, tumor cells in these regions induce the production of hypoxia-inducible factors (HIFs), master transcription regulators that consist of two subunits, the α subunit (HIF-1α, HIF-2α and HIF-3α) and the β subunit (HIF-1β) (Arnt) (1,2). Of these three HIF-α family members, HIF-1α is constitutively expressed, whereas HIF-2α is detected most prominently in vascular endothelial cells during embryonic development and HIF-3α is expressed in kidney and lung epithelial cells (3–5). In addition, although HIF-1β is unaffected by changes in the cellular oxygen concentrations, HIF-1α is O_2_-dependently regulated (1,2,6). Under normoxic conditions, HIF-1α is constantly degraded via the hydroxylation of proline residues within the oxygen-dependent degradation domain (ODD) of HIF-1α by prolyl hydroxylases (PHDs) and the von Hippel-Lindau protein (VHL)-mediated ubiquitin-proteasome pathway. However, under hypoxia, reactive oxygen species (ROS) are generated by mitochondrial electron transport chain and then released to the cytosol, thereby leading to stabilization of HIF-1α through PHD inhibition due to oxidation of Fe^2+^ within PHD (7). The stabilized HIF-1α subunit is translocated into the nucleus, where it forms a heterodimeric transcriptional complex with the HIF-1β subunit and directly binds to the hypoxia-responsive element (HRE, 5′-A/GCGTG-3′) to express a number of its target genes involved in angiogenesis, metabolic adaptation, tolerance of acidosis, cell survival and metastasis, such as vascular endothelial growth factor (VEGF), SLC2A1, which encodes the glucose transporter GLUT1, carbonic anhydrase (CA9), insulin-like growth factor-2 (IGF2) and transforming growth factor-α (TGF-α), respectively (1,8–11). As a result, the expression of HIF-1 facilitates tumor cell survival and growth in hypoxic regions.

Tempol is a member of the family of well-described stable nitroxides that detoxify oxygen metabolites via redox cycling with one-electron transfer reactions and is applied as a standard substance in EPR spectroscopy. As for the biological effects of tempol, its protective effects against radiation-induced alopecia in guinea pigs have been confirmed (12). In addition, the administration of tempol prior to fractionated whole brain radiotherapy resulted in moderate protection against radiation-induced alopecia in a phase I study (13).

In cancer therapy, anticancer drugs and ionizing radiation enhance cell killing effects by targeting DNA in proliferating tumor cells. On the other hand, hypoxic cells show greater resistance to these treatments because these cells display low levels of proliferation in the quiescent state (slow cycling or G0) and exist in the microenvironment where the oxygen effect of ionizing radiation is reduced (14,15). Therefore, hypoxic cells demonstrate a higher possibility of survival after these treatments than normoxic cells in the tumor tissues, potentially resulting in metastasis or recurrence. In other words, treatments targeting hypoxic cells appear to be a promising strategy for eliminating cancer. To date, nitro-imidazole compounds, such as misonidazole, pimonidazole and nimorazole, have been synthesized as hypoxic cell radiosensitizers causing hypoxic tumor cells to be more sensitive to radiation therapy, and these agents have subsequently been tested in clinical trials. Although these drugs exhibit significant radiosensitizing effects *in vitro*, they show low levels of radiosensitization *in vivo* and introduce harmful side effects, including peripheral neuropathy (16). In recent years, bioreductive prodrugs have also been actively developed as a novel hypoxia-targeted drug. In particular, tirapazamine (3-amino-1,2,4-benzotriazine 1,4-dioxide, TPZ), which produces damage to hypoxic cells by ROS produced following one-electron reduction by cytochrome P(450) reductase-enriched microsomes, is currently undergoing evaluation in phase III clinical trials. In addition to those mentioned above, new hypoxia-targeted treatments combined with gene therapy have been developed. For example, Ido *et al* and Harada *et al* showed significant tumor regression and/or growth delay via the selective enhancement of hypoxic cell killing induced by the hypoxia-regulated suicide gene expression using hypoxia-targeted expression vectors harboring the herpes simplex virus type 1 thymidine kinase (HSVtk) and caspase-3 genes under the control of HRE, respectively (17,18).

We found that tempol strongly induced the accumulation of HIF-1α under a combination of hypoxic conditions. This induction mechanism seems to enable us to enhance the hypoxic cell killing by applying the vector bearing the suicide gene fused downstream of HRE. The goal of this study was to evaluate the enhancement of the cell killing effect *in vitro* applying the plasmids that can regulate the suicide gene expression under a combination of tempol and hypoxic conditions and to assess the possibility of its application to gene therapy using tumor-bearing mice boosted with tempol.

## Materials and methods

### Reagent and antibodies

Tempol (4-hydroxy-2,2,6,6-tetramethyl-piperidine 1-oxyl free radical) was purchased from Tokyo Chemical Industry Co., Ltd. (Tokyo, Japan). Apigenin and echinomycin, HIF-1α inhibitors, were purchased from Sigma-Aldrich, Inc. (St. Louis, MO, USA). Anti-HIF-1α antibodies (cat# 3716S), anti-myc-tag antibodies (cat# 2272S) and anti-β-actin antibodies (cat# 4970S) were purchased from Cell Signaling Technology, K. K. (Japan).

### Cell culture and bacteria

All cell lines used in this study, including MCF7 (human breast carcinoma), LNCap (human prostate carcinoma) and Saos2 (human osteoblastic osteo-sarcoma), were grown in RPMI-1640 medium supplemented with 10% (v/v) heat inactivated fetal calf serum, 100 U/ml of penicillin and 100 *µ*g/ml of streptomycin. The cells were incubated in a 5% CO_2_ incubator at 37°C. For hypoxia treatment, the cells were incubated in a hypoxic incubator containing 1.0% oxygen, 5% CO_2_ and 94% nitrogen at 37°C.

The DH5α strain of *Escherichia coli* (*E. coli*) (Takara Bio, Inc., Ohtsu, Japan) was used for the DNA manipulation experiments. The *E. coli* cells were grown in LB medium at 37°C. All medium compositions were purchased from BD Diagnostics (Sparks, MD, USA) and all experiments with *E. coli* were performed according to the methods described by Sambrook and Russell (19).

### Plasmid construction

In order to evaluate the rate of enhancement of the HIF-1α expression induced by tempol treatment under hypoxic conditions, we constructed a plasmid designated p4HRE-Luc-ODD containing the *luc* gene to which the ODD fragment was added under the control of four tandem copies of HRE fragments. To complete the construction of the vector, a plasmid designated p4HRE-Luc was constructed via self-ligation after *Eco*RI digestion of PCR products amplified using pTA-Luc (Takara Bio, Inc.) as a template with the following primers: a forward primer with four copies of HRE consensus sequences, 5′-ATGAATTCTGCACGTACTGCACGTACTGCACGTACTGCACGTAGCGCGTGCTAGCCCGGGCTCG AGA-3′ and reverse, 5′-ATGAATTCTATCGATAGAGAAATGTTCTGGCACCTGC-3′. Underlining indicates HRE consensus sequences (20). A DNA fragment encoding the ODD of HIF-1α (from the 557th to the 574th amino acid of HIF-1α) was amplified using the pBC SK^+^ vector containing cDNA for HIF-1α (cat# ORK01550; Kazusa DNA Research Institute, Kisarazu, Japan) as a template with the following pair of primers, 5′-ATGGTACCGTTAGACTTGGAGATGTT AGCTCCC-3′ and 5′-ATAGAGCTCTAACTGGAA GTCATC ATCCATTGG-3′, and then inserted in the frame at the *Kpn*I and *Sac*I sites created at the 3′ end of the *luc* gene in p4HRE-Luc following digestion of ODD fragments amplified with *Kpn*I and *Sac*I to construct a plasmid designated p4HRE-Luc-ODD. In addition, in order to express a suicide gene under identical regulation to the *luc* gene in p4HRE-Luc-ODD, a plasmid p4HRE-fcy::fur-ODD was constructed by replacing the *luc* gene in the plasmid p4HRE-Luc-ODD with the *fcy::fur* gene, which encodes cytosine deaminase (CD) and uracil phosphoribosyl-transferase (UPRT), amplified using a plasmid pORF5-fcyfur (InvivoGen, San Diego, CA, USA) as a template with the following pair of primers: 5′-ATACTAGTATCACAGAGGAGACCATGGTCACA-3′ and 5′-ATGGTACCGCGACACAGTAGTATCTGTCCCCAAA-3′. The expression of the suicide gene was confirmed by inserting a myc-tag sequence in the frame at the end of the ODD sequence via self-ligation after *Sph*I digestion of PCR products amplified using p4HRE-fcy::fur-ODD as a template with the following primers: forward, 5′-ATGCATGCTAATTCTAGAGTCGGGGCGGCCGG-3′ and reverse, 5′-ATGCATGCTCACAGGTCCTCCTCTGAGATCAGCTTCTGCTCGAGCTCTAACTGGAAGTCATCATCCATT-3′. The orientations and sequences of the constructed plasmids were confirmed using a nucleotide sequencing analysis. Schematic structures for each construct are shown in Figs. 2 and 3.

### Transfection and establishment of stable cell lines

For the transient transfection experiments, 3.0×10^5^ cells were seeded prior to transfection into 60-mm glass Petri dishes and maintained for 12 h in the atmosphere of a 5% CO_2_ incubator at 37°C. In order to determine the rates of enhancement of the HIF-1α activity induced by tempol under hypoxia, the p4HRE-Luc-ODD construct was co-transfected with pGL-4.74, an internal control vector containing the *Renilla luc* gene (Promega, Madison, WI, USA) at a ratio of 50:1 (p4HRE-Luc-ODD vs. pGL-4.70) using the Effectene transfection reagent (Qiagen, Valencia, CA, USA), followed by incubation for 8 h. In addition, the p4HRE-fcy::fur-ODD construct was transfected into MCF7 cells in accordance with the manufacturer’s instructions in order to confirm the expression of the Fcy::Fur-ODD fused protein. We established three stably transfected cell lines. For this process, 1.0×10^6^ MCF7 cells were seeded into 100-mm culture dishes and subsequently transfected with the plasmids p4HRE-Luc-ODD, pGL3-control and p4HRE-fcy::fur-ODD in addition to the plasmid pIRES2-EGFP (Takara Bio, Inc.) containing the neomycin/kanamycin resistance gene. The transfected cells were cultured for ~14 days in culture medium containing 1 mg/ml of G418 (Nacalai Tesque, Kyoto, Japan), after which antibiotic-resistant colonies were isolated and evaluated for the expression of the gene of interest (Luc-ODD, Luc or Fcy::Fur-ODD) in order to select successfully established stable transfectants. Representative colonies were proliferated and designated the MCF7/HRE-Luc-ODD, MCF7/SV40-Luc or MCF7/HRE-fcy::fur-ODD cell lines, respectively.

### Luciferase reporter assay

Following transfection, the cells were incubated for 12 h in fresh medium and then subjected to various combination treatments with tempol and O_2_ at different durations of incubation. As for the HIF-1α inhibition experiments with apigenin, the transfected cells were treated with 40 *µ*M of apigenin or vehicle [0.1% dimethylsulfoxide (DMSO)] for 1 h prior to exposure to the hypoxic conditions. Echinomycin was also used as an inhibitor for HIF-1α in a similar manner. The treated cells were then washed in phosphate-buffered saline (PBS) and lysed with 400 *µ*l of passive lysis buffer (Promega) for 15 min at an ambient temperature. A Luc assay was performed using Dual-Luciferase assay reagent (Promega), in accordance with the manufacturer’s instructions. The Luc activity of the p4HRE-Luc-ODD construct was determined in relative luminescence units (RLU), where the value of luminescence by the firefly Luc activity was divided by that of the *Renilla* Luc activity in the same lysate. The degree of enhancement of the Luc activity induced by each treatment was expressed as the fold induction, where the RLU value for a sample treated with a given treatment was divided by that for an identically prepared sample treated without the treatment.

### Western blot analysis

Following the various treatments, 1.5×10^6^ cells were washed in PBS twice and harvested via centrifugation. The cells were then lysed in 150 *µ*l of RIPA buffer [50 mM Tris-HCl pH 7.4, 400 mM NaCl, 1% (v/v) Nonidet P-40 and 0.25% (w/v) Na-deoxycholate] with protease inhibitor (Sigma-Aldrich) and stored in a freezer at −20°C until use. The cell lysates (40 *µ*g/lane) were subsequently separated using 4–20% gradient polyacrylamide with SDS-polyacrylamide gel electrophoresis and transferred onto nitrocellulose membranes (Schleicher & Schuell, Keene, NH, USA). After blocking the membranes with 3% skim milk in PBS for 1 h, the cells were incubated with anti-HIF-1α antibodies (1:500), anti-Myc-tag antibodies (1:1,000) or anti-β-actin antibodies (1:1,000) overnight at 4°C. After washing the membranes three times with 0.1% Triton X-100 in PBS, the cells were incubated with horseradish peroxidase-conjugated secondary antibodies for 90 min, and the protein expression was visualized with ECL and blotting detection reagents using an LAS-500 luminescence imaging analyzer (all from GE Healthcare, UK Ltd., Buckinghamshire, UK).

### Colony formation assay

MCF7/HRE-fcy::fur-ODD cells were plated into culture dishes and exposed to medium containing 2 mM tempol, 100 *µ*M of CoCl_2_ and 10 mM 5-fluorocytosine (5-FC) for 48 h. After replacing the medium in the dishes with fresh medium, the cells were incubated to form colonies for 14 days. For the evaluation, the formed colonies were stained with methylene blue and surviving colonies consisting of more than ~30 cells were counted. The plating efficiency (PE) was defined as the number of observed colonies divided by the number of plated cells treated without any treatment. The surviving fraction (SF) was calculated as the number of observed colonies divided by the number of plated cells after treatment, with correction using the PE.

### Luc activity in the tumor tissues

Suspensions of 3.5×10^6^ MCF7/HRE-Luc-ODD and MCF7/SV40-Luc cells in PBS were mixed with an equal volume of Matrigel Basement Membrane matrix (BD Biosciences, Bedford, MA, USA) and subcutaneously injected into the left and right flanks of 4-week-old KSN mice separately. When the tumors grew to 10 mm in average diameter after inoculation, the tumor-bearing mice were subjected to *in vivo* bioluminescence experiments. For the control experiment, the mice were injected intra-peritoneally with 500 *µ*l of tempol at 100 mM in PBS or PBS alone. For *in vivo* bioluminescent imaging, the tumor-bearing mice were injected with Luciferin EF (Promega) at a dose of 100 *µ*g/g body weight intraperitoneally 6 h after tempol or PBS administration and then subjected to treatment with a bioluminescence detection system (AEQUORIA-2D/c8600; Hamamatsu Photonics K.K., Hamamatsu, Japan) 5 min after substrate administration. Images of the Luc expression were captured with integration time for 60 sec using the Wasabi application software program (ver. 1.5; Hamamatsu Photonics K.K.). The Luc activity was determined in RLU, where the luminescence value of the MCF7/HRE-Luc-ODD tumor was divided by that of the MCF7/SV40-Luc tumor in a given mouse. The degree of enhancement of the Luc activity induced by tempol in each tumor was expressed as the ratio of RLU, where the RLU value after tempol injection was divided by that observed before tempol injection.

### Statistical analysis

All values are expressed as the mean ± standard deviation. Significant differences between groups were determined using a one-way analysis of variance (ANOVA) or the Student’s unpaired t-test. If the results of the ANOVA were significant, the Bonferroni/Dunn procedure was used as a post hoc test. A P<0.05 was considered to be statistically significant.

## Results

### Tempol strongly enhances the expression of HIF-1α in combination with hypoxia or CoCl_2_ treatment

Tempol is currently being assessed in a Phase II clinical trial as a drug to prevent radiation-induced alopecia. However, little is known about its detailed effects on the gene expression profiles. We thus examined the influence of tempol on the accumulation of HIF-1α using a western blot analysis. Among the genes tested, the expression of HIF-1α, which plays an essential role in cellular responses to hypoxia, was markedly increased in the MCF7 cells by treatment with 2 mM tempol and 1.0% O_2_ for 6 h (Fig. 1). The strongly enhanced HIF-1α expression was observed 24 h after incubation with tempol under conditions of hypoxia (data not shown). Similarly, treatment with 100 *µ*M CoCl_2_, a hypoxia-mimicking agent, enhanced the expression of HIF-1α in combination with the application of 2 mM tempol. Meanwhile, the HIF-1α expression was detected at very low levels when the cells were treated with tempol under normoxia (Fig. 1). These results indicate that tempol selectively enhances the HIF-1α expression under conditions of hypoxia.

We next carried out a Luc reporter assay to evaluate the degree of enhancement of the activity of HIF-1α induced by combination treatment with tempol and hypoxia. A plasmid, p4HRE-Luc-ODD, containing the *luc* gene linked to four tandemly repeated HRE/TATA boxes and a DNA fragment with the ODD sequence was constructed and transiently transfected into MCF7 cells (Fig. 2A). Consequently, the Luc activity in the cells transfected with p4HRE-Luc-ODD treated under 1.0% O_2_ for 6 h was ~22-fold that observed in the control cells under normoxia, while the Luc activity in the cells transfected with p4HRE-Luc-ODD treated with 2 mM tempol under 1.0% O_2_ increased up to ~217-fold compared to that noted in the no tempol-treated cells under normoxia (~10-fold enhancement compared to that in the no tempol-treated cells under 1.0% O_2_; P<0.001, Fig. 2B). Similarly, the expression of HIF-1α in the cells treated with both 2 mM tempol and 100 *µ*M of CoCl_2_ demonstrated much higher enhancement (~181-fold) than that noted in the no tempol-treated cells under normoxia (P<0.001, Fig. 2B). However, the transfected cells treated with more than 2 mM tempol showed a lower Luc activity than the no tempol-treated cells and high cytotoxicity associated with alteration of their cell shape. In order to obtain more detailed data regarding the enhancement of HIF-1α by tempol, we assessed the O_2_ concentration- and time-dependent effects in enhancing the HIF-1α expression. For the O_2_ concentration-dependent effects study, transient cells were exposed to medium containing O_2_ at various concentrations (0.5, 1.0, 3.0 or 5.0%) with 2 mM tempol for 6 h. As shown in Fig. 2C, the degree of enhancement of the HIF-1α expression in the no tempol-treated cells was highest at 0.5% O_2_ and decreased as the O_2_ concentration increased. In contrast, the extent of enhancement of the HIF-1α expression in the tempol-treated cells was highest at 1.0% O_2_, indicating a different pattern from that observed in the no tempol-treated cells. These results were also confirmed by western blot analysis (data not shown). As for the time-dependent effects study, enhancement of the HIF-1α expression in the cells treated with tempol under 1.0% O_2_ was observed at 3 h and peaked at 6 h, then gradually declined thereafter, as shown in Fig. 2D. Moreover, the expression of HIF-1α in these cells showed much greater enhancement (157- to 267-fold) at all incubation times than that observed in the cells treated with either tempol alone or hypoxia alone (Fig. 2D).

We then confirmed whether the expression levels of HIF-1α in the other cell lines were also affected by treatment with tempol under conditions of hypoxia. Consequently, LNCaP cells and Saos2 cells were subjected to similar assays. Following treatment with tempol, the HIF-1α expression levels in the two cell lines under hypoxia were significantly enhanced compared to that observed in the two cell lines exposed to identical conditions with the exception of tempol treatment (Fig. 2E). However, the degree of enhancement of the HIF-1α expression induced by tempol treatment in the Saos2 cells at 1.0% O_2_ was ~10 times less than that noted in the MCF7 or LNCap cells, suggesting the presence of cell type-dependent variation in the level of HIF-1α enhancement induced by tempol.

In order to verify that the increase in the Luc activity of p4HRE-Luc-ODD after the combined treatment with tempol and hypoxia was caused by the enhanced HIF-1α expression, we performed experiments employing an inhibitor of the HIF-1 expression, apigenin. As a result, the addition of apigenin significantly suppressed the induction of the Luc activity of p4HRE-Luc-ODD in the MCF7 cells treated with 2 mM tempol under hypoxia by up to 86%, confirming an HIF-1α-dependent increase in Luc activity (Fig. 2F). We then conducted similar experiments using echinomycin, an inhibitor of the binding of HIF-1 to HRE. In the presence of this inhibitor, the increase in the Luc activity induced by tempol in the cells transfected with p4HRE-Luc-ODD under hypoxia was suppressed in a concentration-dependent manner (data not shown). Based on these results, we conclude that the enhancement of the Luc activity caused by the enhancement of HIF-1α and tempol treatment strongly enhances the expression of HIF-1α in combination with hypoxia or CoCl_2_ treatment.

### Selective enhancement of hypoxic cell killing with the tempol-regulated suicide gene expression

The phenomenon in which the expression of HIF-1α is enhanced by treatment with tempol under hypoxia may be applied to selectively enhance cell killing under hypoxia. In order to test this hypothesis, we constructed a plasmid, p4HRE-fcy::fur-ODD, by replacing the *luc* gene of p4HRE-Luc-ODD with a suicide gene, the *fcy::fur* gene (Fig. 3A). The suicide gene was similarly modified in terms of the ODD sequence with a myc-tag sequence attached at the end. The *fcy::fur* fusion gene product exhibits a CD and UPRT activity, which efficiently converts the less cytotoxic 5-FC to the highly cytotoxic 5-FU and 5-FUMP. Therefore, cells expressing this gene are killed in the presence of 5-FC. As shown in Fig. 3B and C, enhancement of the *fcy::fur* fusion gene expression by tempol under hypoxia was verified by western blot analysis using antibodies against myc-tag. Moreover, strongly enhanced expression levels of the *fcy::fur* fusion gene product were observed in both cells transiently and stably transfected with MCF7/HRE-fcy::fur-ODD when treated with tempol under hypoxia. A similar tendency was observed among the stably transfected cells cultured with CoCl_2_ instead of under hypoxia. These results are consistent with those obtained in the Luc reporter assay described above, indicating that the *fcy::fur* fusion gene expression is also enhanced by tempol, similar to the *luc* gene.

We then carried out a colony formation assay to evaluate the degree of enhancement of selective cell killing induced by tempol under hypoxic mimic conditions using MCF7/HRE-fcy::fur-ODD cells. Stably transfected cells were cultured in the presence of 2 mM tempol and 100 *µ*M of CoCl_2_ in addition to 10 mM 5-FC for 48 h, and the cultured cells were washed in fresh medium and further incubated without these chemicals for ~2 weeks to allow the cells to form colonies. The number of colonies formed by the tempol-treated cells was much lower than that formed by the control cells, even without 5-FC treatment, suggesting that these effects were possibly due to the cytotoxicity of tempol. On the other hand, when stably transfected cells were cultured in medium containing all of the chemical reagents of tempol, CoCl_2_ and 5-FC, the number of colonies was significantly reduced by 19-fold compared to that formed by the cells treated similarly with the exception of 5-FC (Fig. 4A and C). In addition, alteration of the cellular morphology was observed only when the cells were cultured in medium containing all of the chemical reagents (Fig. 4B). These results suggest that the application of this suicide gene expression regulation system composed of an HRE promoter and the ODD sequence in combination with tempol treatment may be useful for the selectively killing of cells under hypoxia.

### Enhancement of the HIF-1α expression by tempol in the solid tumors

Hypoxic regions have been reported to be found inside solid tumor tissues. We thus investigated whether the gene expression system developed in this report can be applied for gene regulation in hypoxic regions of solid tumors *in vivo*. We subsequently examined changes in the Luc activity in the xenograft MCF7/HRE-Luc-ODD and MCF7/SV40-Luc tumor tissues in nude mice following the injection of tempol by observing the extent of photon generation due to the oxidation of a substrate administered to the mice. As shown in Fig. 5, the ratio of RLU in the mice injected with tempol was increased by more than 2.8±1.9 times compared with that observed in the control group injected with PBS, suggesting the regulation of the gene expression by our system following tempol injection both *in vivo* and *in vitro*. However, the fold induction observed *in vivo* was much lower than that obtained *in vitro*.

## Discussion

In the present study, we demonstrated the effects of tempol in upregulating the HIF-1α expression directly as well as indirectly via an increase in the Luc expression of p4HRE-Luc-ODD. Furthermore, under hypoxic conditions, it was confirmed that tempol upregulated the *luc* gene expression of p4HRE-Luc-ODD in all three transfected cell lines employed in this study (MCF7, LNCap and Saos2), although to various degrees. Notably, all of these episodes of upregulation were suppressed by treatment with either apigenin, an inhibitor of the HIF-1 expression, or echinomycin, an inhibitor of the binding of HIF-1 to HRE, thus confirming that tempol upregulated the Luc expression via upregulation of the HIF-1α expression. Considering the expression of the *luc* gene under the control of four copies of HRE in the p4HRE-Luc-ODD transfected MCF7 cells as an index of HIF-1α activity, the HIF-1α expression was inversely regulated according to the oxygen concentration. Namely, the rate of induction reached a maximum at an oxygen concentration of 0.5%, the minimum applied in this study, and subsequently declined in an exponential manner as the oxygen concentration increased. On the other hand, when the cells were treated with tempol, the rate of induction reached a peak at an oxygen concentration of 1.0% rather than 0.5% (Fig. 2C). The p4HRE-Luc-ODD construct carries a promoter composed of four copies of HRE and the TATA-box to drive the *luc* gene. Therefore, the expression of this gene is tightly controlled by the HIF-1α expression. In other words, it inversely correlates with the oxygen concentration. In addition, the Luc protein attaches with the ODD domain at its C-terminal end, such that its accumulation is also inversely regulated based on the oxygen concentration. Therefore, oxygen suppresses the transcription of the *luc* gene and the accumulation of Luc proteins in our gene regulation system applied for p4HRE-Luc-ODD. However, the Luc expression was the highest at 1.0% oxygen concentration, rather than 0.5%, when MCF7 cells transiently transfected with p4HRE-Luc-ODD were treated with tempol, suggesting that the upregulation of HIF-1α is not necessarily dependent on the degree of hypoxia. Although the reason for this observation remains unknown, we consider that the expression of the luc gene in our gene regulation system may be determined by the balance between the increase in the HIF-1α expression achieved with tempol treatment and the degradation of HIF-1α and Luc via ODD induced by oxygen.

We then applied our gene regulation system for cancer gene therapy targeting hypoxic regions using the *fcy::fur* fusion gene that converts 5-FC, a pro-drug, to 5-FU, an anticancer drug as a suicide gene. Consequently, the rate of cell survival in the MCF7/HRE-fcy::fur-ODD cells treated with tempol under normoxia was not affected by the addition of 5-FC, suggesting that the cell death observed under these conditions was due to the cytotoxicity of tempol. In contrast, when these cells were treated with 5-FC in the presence of tempol and CoCl_2_, a hypoxic mimic compound, a 19-fold higher cell death rate was observed compared with that noted in the same cells treated identically with the exception of 5-FC. These results indicate that our gene regulation system increased the suicide gene expression in response to the addition of tempol only under hypoxia, thereby facilitating cell killing specifically in hypoxic regions. Interestingly, the rate of cell killing in the stably transfected cells treated with tempol and CoCl_2_ only in the absence of 5-FC was much lower than that observed in the same cells treated identically with the exception of CoCl_2_. Although the precise reasons for this phenomenon remain unclear, we assume that the oxidized form of tempol is converted to its reduced form via a reaction with cobalt, presumably reducing the cytotoxicity of tempol.

Furthermore, we performed an *in vivo* experiment to evaluate whether our gene regulation system works *in vitro* in order to explore possible applications for cancer gene therapy. We prepared two cell lines: MCF7/HRE-Luc-ODD and MCF7/SV40-Luc. The former cell line was stably trans-fected using our gene regulation system to express the *luc* gene in response to tempol under hypoxia, while the latter was stably transfected using a control gene expression system to express the *luc* gene under the control of the strong SV40 promoter, which is not affected by either tempol or hypoxic conditions. Mice were subcutaneously administered the former cell line in the right flank and the latter cell line in the left flank. Following tumor formation, using an *in vivo* imaging apparatus, we evaluated the increase in the Luc expression based on the degree of luminescence emitted via the oxidation of a substrate injected intraperitoneally before and after tempol stimulation. The amount of luminescence emitted from the MCF7/HRE-Luc-ODD tumors in the mice administered tempol was 2.8 times higher than that emitted from the same tumors in the mice administered PBS. Although this difference was statistically significant (P=0.0141), it was very small compared to that observed in the *in vitro* experiment. Tempol is a stable free radical of organic matter with an unpaired electron. Based on the obtained results, the HIF-1α expression is upregulated by the oxidized form of tempol. In the living body, the oxidized form of tempol is converted to the reduced form by antioxidants, including glutathione. Hyodo and colleagues reported the period of the conversion from the oxidized forms to the reduced forms in the living body to be 2–3 min (21). In addition, hypoxic regions in tumor tissues are located 70–100 mm from blood vessels (22). Hence, in the living body, the access of tempol to hypoxic regions is hampered by its short-lived activity and the long distance from blood vessels. We consider one reason for the smaller degree of HIF-1α enhancement observed in this study to be that the number of molecules having an effect on the HIF-1α expression *in vivo* is fewer than that seen *in vitro*, thus reducing the rate of enhancement of the Luc expression in the tumor xenograft model. Furthermore, the pressure of oxygen in solid tumors is known to be highly heterogeneous, with the overall hypoxic fraction (pO_2_ ≤2.5 mmHg) in tumors estimated to be <25% according to clinical studies employing computerized polarographic needle electrodes (23). Therefore, it is difficult to detect the chemiluminescence of the Luc expression due to the significantly reduced numbers of hypoxic cells in the tumor tissues versus *in vitro* experiments, resulting in smaller levels of enhancement of HIF-1α in the living body. Considering the application of our system, which regulates the suicide gene expression in hypoxic regions, for site-specific cancer gene therapy, nitroxides with similar properties to tempol, including high membrane permeability and a longer period of being in the oxidized form in the living body, may be the ideal compound to regulate suicide gene expression in hypoxic environments, if it is less cytotoxic.

Hypoxic cells show resistance to radiation therapy and chemotherapy due to the ability of a fraction of these cells to survive after therapy, thus remaining a source for recurrence and metastasis. Therefore, there have been many attempts to target hypoxic cells. Among such approaches, gene therapy for only hypoxic regions has been developed, in which a suicide gene is expressed under the control of HRE to specifically target cells in hypoxic regions. However, with current technology, it is very difficult to transfer an adequate vector to eradicate all hypoxic cells. Therefore, our method of enhancing the suicide gene expression specifically in hypoxic regions using nitroxide is a promising strategy for targeting hypoxic cells.

## Figures and Tables

**Figure 1:** Tempol strongly induces the accumulation of the HIF-1α in combination with hypoxia or CoCl_2_ treatment. MCF7 cells were exposed to hypoxia (1.0% O_2_) or normoxia with or without 2 mM tempol for 6 h and harvested for western blot analysis of the HIF-1α protein. The same experiments were also performed in the presence of 100 *µ*M CoCl_2_. β-actin served as the loading control for the western blot analysis. HIF, hypoxia-induced factor.

**Figure 2:** HIF1α-inducible properties induced by tempol under various conditions. (A) Schematic structure of the reporter plasmid p4HRE-Luc-ODD. The promoter sequence consisted of four copies of HRE fragments and the TATA-box was fused upstream of the *luc* gene. The ODD sequence amplified from HIF1α cDNA was inserted downstream of this site. (B) Induction of the Luc activity by tempol under hypoxia or CoCl_2_ treatment. MCF7 cells transiently transfected with the plasmid p4HRE-Luc-ODD were allowed to recover for 12 h after transfection under normoxia and exposed to hypoxia (1.0% O_2_) or treated with 100 *µ*M of CoCl_2_ with or without 2 mM tempol for 24 h and then assayed for Luc activity. The fold induction was calculated by dividing the RLU of each stimulated cell by the RLU of the control cells under normoxia without tempol. Each column presents the average and standard deviation (n=5–7). ^**^P<0.001, significant increase vs. hypoxia and CoCl_2_ without tempol (ANOVA with Bonferroni/Dunn). (C) Induction of the Luc activity in the transiently transfected MCF7 as a function of the oxygen concentration. The transfected cells were exposed to various concentrations of O_2_ (0.5, 1.0, 3.0 and 5.0% O_2_) with or without 2 mM tempol for 24 h. The fold induction was calculated by dividing the RLU of the transfected cells with or without tempol at various O_2_ concentrations by the RLU of the control cells under normoxia without tempol. The error bars represent the standard deviation (n=5). (D) Time courses of the Luc activity induced by tempol under hypoxia and normoxia. The transfected MCF7 cells were exposed to 1.0% O_2_ or normoxia with or without 2 mM tempol, and the fold induction was calculated by dividing the RLU of each stimulated cell by the RLU of the control cells under normoxia without tempol at the indicated time-points (3, 6, 12 and 24 h). The error bars represent the standard deviation (n=5). (E) Induction of the Luc activity in three cancer cell lines, MCF7, LNCap and Saos2, by tempol under hypoxia and normoxia. Each cell line was exposed to 1.0% O_2_ with 2 mM tempol for 24 h. The fold induction was normalized to the RLU of the control cells treated without tempol under normoxia. Each column presents the average and standard deviation (n=3–7). ^*^P<0.05 and ^**^P<0.01, significant increase vs. hypoxia (ANOVA with Bonferroni/Dunn). (F) Suppression of the Luc activity by HIF!1α, apigenin. The transfected cells were treated with 40 *µ*M of apigenin or vehicle (0.1% DMSO) for 1 h prior to exposure to 1.0% O_2_ with or without 2 mM tempol for 24 h. The fold induction was normal-ized to the RLU of the control cells treated without tempol and apigenin under normoxia. Each column presents the average and standard deviation (n=5–7). ^**^P<0.01, significant increase vs. without apigenin (ANOVA with Bonferroni/Dunn). HIF, hypoxia-induced factor; ODD, oxygen-dependent degradation domain; HRE, hypoxia-responsive element; RLU, relative luciferase units.

**Figure 3:** Tempol enhances the expression of the suicide gene, the *fcy::fur* fusion gene, in combination with hypoxia or CoCl_2_. (A) Schematic structure of the suicide gene, the *fcy::fur* fusion gene, regulated by four copies of HREs and ODD under hypoxia. The plasmid p4HRE-fcy::fur-ODD for gene therapy was constructed by replacing the *luc* of the plasmid p4HRE-Luc-ODD with the *fcy::fur* fusion gene. The myc-tag was inserted at the C-terminal of the Fcy::Fur-ODD to identify the expression of the fusion proteins in the transfected cells. (B) Western blot analyses of the Fcy::Fur fusion proteins demonstrated enhancement in both the transient and stable expression clones, MCF7/HRE-fcy::fur-ODD, in combination with 2 mM tempol and hypoxia treatment (1.0% O_2_) for 24 h. (C) Western blot analyses of the Fcy::Fur fusion proteins enhanced by tempol under treatment with 100 *µ*M of CoCl_2_ for 24 h. β-actin served as a loading control for western blotting. ODD, oxygen-dependent degradation domain; HRE, hypoxia-responsive element.

**Figure 4:** Selective enhancement of hypoxic cell killing by Fcy::Fur fusion proteins induced by treatment with a combination of tempol and CoCl_2_. (A) Selective hypoxic cell killing was assessed using a colony formation assay. After the stable expression clone, MCF7/HRE-fcy::fur-ODD cells, was treated with 2 mM tempol and 100 *µ*M of CoCl_2_ for 48 h in 10 mM 5-FC-containing medium, the cells were divided and plated for a colony formation assay for 14 days. 5-FC (-), colony incubated without 5-FC; 5-FC (+), colony incubated with 5-FC. (B) Alteration of the cellular morphology of the stable cell lines treated with 2 mM tempol and/or 100 *µ*M of CoCl_2_ in 5-FC-containing medium. (C) Surviving fraction of the stable expression clone, MCF7/HRE-fcy::fur-ODD, after treatment with 2 mM tempol and/or 100 *µ*M of CoCl_2_. The error bars represent the standard deviation (n=3). ^**^P<0.01, significance vs. without 5-FC (Student’s unpaired t-test). ODD, oxygen-dependent degradation domain; HRE, hypoxia-responsive element.

**Figure 5:** Enhancement of the HIF-1α activity in the tumors of living mice induced by tempol. The stable expression clone, MCF7/HRE-Luc-ODD or MCF7/SV40-Luc, was implanted into the legs of the mice. The tumor-bearing mice were injected intraperitoneally with 100 mM tempol and fasted for 6 h, after which the *in vivo* bioluminescence emitted from the tumors was measured 3 min after the injection of D-luciferin. The error bars represent the standard deviation (n=3). ^*^P<0.05, statistical significance vs. PBS (Student’s paired t-test). HIF, hypoxia-induced factor; ODD, oxygen-dependent degradation domain; HRE, hypoxia-responsive element.

## Abbreviations

HIF: hypoxia-inducible factor
Luc: luciferase
ODD: oxygen-dependent degradation domain
HRE: hypoxia-responsive element
PHD: prolyl hydroxylase
VHL: von Hippel-Lindau protein
ROS: reactive oxygen species
VEGF: vascular endothelial growth factor
GLUT: glucose transporter
CA: carbonic anhydrase
IGF: insulin-like growth factor
TGF: transforming growth factor
TPZ: tirapazamine
HSVtk: herpes simplex virus type 1 thymidine kinase
RLU: relative luciferase units
CD: cytosine deaminase
UPRT: uracil phosphoribosyltransferase
